This article has been retracted.

# A Diagnostic Scoring System for Distinguishing between Tuberculous and Bacterial Meningitis Based on Clinical and Laboratory Findings

**DOI:** 10.1155/2021/1220650

**Published:** 2021-07-27

**Authors:** Hongyan He, Yueli Zou, Junying He, Hui Bu, Yaling Liu

**Affiliations:** ^1^Department of Neurology, The Second Hospital of Hebei Medical University, Shijiazhuang, Hebei, China; ^2^Neurological Laboratory of Hebei Province, Shijiazhuang Hebei, China; ^3^Institute of Cardiocerebrovascular Disease, Shijiazhuang Hebei, China; ^4^Department of Neurology, Hebei Chest Hospital, Shijiazhuang, Hebei, China

## Abstract

It is very difficult to diagnose and distinguish tuberculous meningitis, and the current laboratory methods are unsubstantial in developing countries. The study is aimed at creating a scoring system on the basis of basic laboratory and clinical achievements that could be used as diagnostic aid for tuberculous meningitis for Chinese patients. A retrospective study of cases was conducted for comparison between clinical characteristics and laboratory features of 241 patients on admission who conformed to inclusion criteria of tuberculous meningitis (*n* = 141) or bacterial meningitis (*n* = 100). Logistic regression was employed to establish a diagnostic formula to distinguish between tuberculous meningitis and bacterial meningitis. The receiver operating characteristic curve analysis was applied to determine the best diagnostic critical point of the diagnostic formula. It was found that five variables (disease course, white blood cell count, serum sodium, total white cell count of cerebrospinal fluid, and neutrophil proportion in cerebrospinal fluid) were independently associated with tuberculous meningitis. The 87% sensitivity and 94% specificity were included in the diagnostic scoring system derived from these variables. Especially in the case of limited microbial resources, doctors can use this diagnostic scoring system to distinguish tuberculous meningitis from bacterial meningitis.

## 1. Introduction

Tuberculous meningitis (TBM) still is regarded as a common infection in the central nervous system (CNS), especially in areas, such as China, where have a high prevalence of tuberculosis. TBM is regarded as the most severe infection for mycobacterium tuberculosis (MTB) and has significant morbidity and mortality in both adults and children [1–3]. Despite antituberculosis chemotherapy, more than 50% of patients die or develop into serious neurological sequelae due to late diagnosis [4]. It is regarded that the most important prognostic factors are early diagnosis and treatment of TBM. Isolation of MTB from the cerebrospinal fluid (CSF) is critical for the diagnosis of definite TBM. Nevertheless, current microbiological diagnosis and molecular assays lack sufficient sensitivity. As for smear microscopy of CSF using Ziehl–Neelsen (ZN) staining, CSF culture, and GeneXpert MTB/RIF (Xpert), detection of MTB that was found in TBM patients' paucibacillary CSF is difficult [5]. Therefore, clinicians must depend on the clinical features, laboratory findings, and imaging manifestations for appropriate diagnosis and treatment. Unfortunately, clinical manifestations and biochemical features in CSF of TBM are similar to other infections of CNS, especially bacterial meningitis (BM) which is partially treated. In several studies, authors have tried to describe clinical features and laboratory parameters which are predictive in the early diagnosis of TBM via applying logistic regression to build a diagnostic method, particularly suitable for areas where tuberculosis is common and limited resources are issues [6–8]. However, there are few relevant diagnostic methods for distinguishing tuberculous meningitis from bacterial meningitis. Therefore, this study intended to develop a diagnostic scoring system based on clinical data and laboratory achievements that could be taken as a predictor of TBM in China.

## 2. Objects and Methods

### 2.1. Objects

A total of 241 patients with CNS infection admitted to the neurology ward of the Second Hospital of Hebei Medical University from January 2010 to December 2016 were selected as the research subjects, including 155 males and 86 females. The age range of the patients was 23~51 years old, with the average age of 32.45 ± 2.96 years. All subjects included in the study were divided into a TBM group (141 cases) and a BM group (100 cases) based on the diagnosis results. All patients in the neurology ward of our hospital with CNS infection were evaluated based on the diagnostic criteria of TBM and BM. TBM patients with microbiological confirmation were included in the further study. The inclusion criteria of BM were applicable for those with confirmed or clinical BM (partly treated BM). The exclusion criteria of this study were defined as follows: patients with unclear diagnosis results, patients with incomplete case data, patients with TBM retreatment, and patients whose course of disease was more than 1 month. The research process had been approved by the ethics committee of the hospital, and all subjects included in the study had signed the informed consent forms.

### 2.2. Diagnostic Criteria

The TBM diagnosis was classified into “definite,” “probable,” and “possible” based on the case definition put forward by Marais et al. [9]. Marais et al. figured out a diagnostic scoring system, including four sections about evaluation of clinical characteristics, CSF findings, cerebral imaging, and evidence of tuberculosis outside the CNS (Table 1). Definite TBM was made by the following criteria: smear microscopy for acid-fast bacilli (AFB) shown in CSF or MTB which were cultured in CSF or a commercial positive MTB nucleic acid amplification test. Patients were probable TBM if the total score was at least 12 (when cerebral imaging was difficult to get, the total score decreased to at least 10), while it was compatible between patients who got the score of 6–11 and who were possible TBM (if cerebral imaging was unavailable, the score decreased to 6–9), having the lowest 2 points of CSF or cerebral imaging criteria [10].

The diagnosis of BM was made by the following criteria: (1) pathogenic bacteria were separated from the CSF or (2) clinical meningitis including the following: lymphocytes and neutrophils and low glucose concentration in the CSF (<50% in blood), sterile blood and CSF cultures, and full recovery when no one accepted antituberculosis chemotherapy within 3 months after admission [6, 7].

### 2.3. Disease Severity

The classification of neurological stages of patients was made according to the modification of the British Medical Research Council (BMRC) definition—stage I: 15 points in the Glasgow Coma Scale (GCS) without focal neurologic signs; stage II: the GCS score of 11–14 or with meningeal irritation, slight or no conscious modification, and minor neurological impairment (such as cranial nerve palsy); and stage III: severe conscious modification, seizure, and focal neurological deficit (GCS score < 10) [11–13].

### 2.4. Statistical Analysis

A comparison was made about the 30 clinical data and laboratory parameters of patients who met the inclusion criteria of TBM and BM. The analytical methods were applied to determine the normality of the continuous variables (Kolmogorov-Smirnov test). Results were expressed by the median and interquartile range of continuous variables and frequency (%) of categorical variables.

Comparison was made about variables between the two groups via the univariate Analysis. Mann–Whitney *U*-test and chi-square test were applied to study continuous and categorical variables, respectively. Variables which are statistically significant between two groups were analyzed in the multivariate logistic regression to test independent predictors of TBM. The receiver operating characteristic curve (ROC) was employed to find the best diagnostic segmentation point of continuous variables and convert them into dichotomous variables. At the same time, the logistic regression analysis was applied to build a diagnostic model. The diagnostic index (DI) of each clinical variable in the model was defined by relying on rounded *β*-coefficients of the model. The total diagnostic index (TDI) was calculated by aggregating all variable DIs, TDI = DI (disease course exceeding 4.5 days) + DI (white blood cell count of less than less than 12.15 × 109/L) + DI (serum sodium of less than 132.8 mmol/L) + DI (total CSF white cell count of less than 499 × 103/mL) + DI (the neutrophil proportion in CSF of less than 59%). TDI was defined as a diagnostic scoring system about a differential diagnosis between TBM and BM. It was found that the optimum segmentation point for the TDI was 6 depending on the ROC. TBM was confirmed when TDI was equal to or greater than 6; and BM was confirmed when TDI < 6. The ROC was applied to get the optimum segmentation of the combined diagnostic indices. All analyses had results of SPSS 22. It was statistically significant with a *P* value < 0.05. Meanwhile, results got odds ratio and 95% confidence interval.

## 3. Results

A total of 384 patients meeting the diagnostic criteria participated in our study. Wherein, 284 patients were diagnosed as TBM and 100 patients were BM. Among TBM patients, 141 were categorized as definite TBM, 44 probable TBM, and 99 possible TBM. MTB was isolated from the CSF of 141 patients, 27 cases were positive by ZN and Xpert, 108 cases were positive by ZN alone, and 6 cases were positive by Xpert alone. Bacterial pathogen was isolated from the CSF of 20 patients. A further 80 adults, including those partly treated, satisfied the clinical diagnostic criteria for BM. We compared clinical and laboratory results about 141 definite TBM patients with those of the 100 patients with BM.

The univariate analysis revealed that it was significantly different between two groups in the terms of parameters, including sex, disease course, recent loss of weight, night sweats, meningeal signs, cranial nerve palsies, WBC, the neutrophil proportion, HCT, serum sodium, CSF/blood glucose, clear appearance of CSF, total count of CSF WBC, neutrophil proportion in CSF, and CSF chloride (Table 2).

It was found that six variables (disease course, WBC, neutrophil proportion in blood, serum sodium, total CSF white cell count, and neutrophil proportion in CSF) were independently correlated with the diagnosis of TBM by applying the logistic regression analysis (Table 3).

There was a conversion from continuous variables to categorical variables according to the optimal separation generated by the ROC curve. Multivariate analysis was performed to construct a diagnostic rule. Five variables were present in the final diagnostic model (Table 4).  Table 5 showed the DI for five variables.

The diagnostic sensitivity and the diagnostic specificity were 87% and 94%, respectively. Area under ROC curve (AUC) = 0.962 (Figure 1).

## 4. Discussion

There are many difficulties and challenges in the diagnosis of TBM. Prognosis can be improved relying on early identification and appropriate antitubercular therapy. In our study, the vast majority of patients (59%) with definite TBM were classified as stage III, whereas only 8% patients presented to be in stage I. The late presentation was most likely due to the delayed referral to the tertiary centers. In addition, most patients were from rural areas, where the health care facilities were limited.

As for diagnosis of TBM, isolation of MTB from CSF has been regarded as the gold criterion. The sensitivity of CSF microscopy is about 10%–20%. There are evidences that show that the sensitivity may depend on the examination volume of CSF, the time taken over microscopy, the speed, and the duration of centrifugation, but it rarely exceeds 60% [14]. The sensitivity of the culture of MTB from CSF is more sensitive than CSF microscopy. But a biosafety level 3 laboratory is required in the CSF culture, ideally. CSF culture is time-consuming because liquid media culture and solid media culture need at least 10 days and 8 weeks, respectively [15]. As for clinical decision-making, CSF culture was too slow and few hospitals have the required facilities. The development of nucleic acid-based amplification tests to detect MTB-specific molecules was limited due to insensitivity and long term of conventional bacteriology. Xpert was recognized by the World Health Organization (WHO) in 2010, and this assay is currently being recommended as a preferred initial diagnostic test. Several studies had investigated the function of Xpert in the diagnosis of TBM. The sensitivity and specificity of this method were found to be about 60% and close to 100% [16–18]. Unfortunately, the facility was expensive and it was difficult to carry out the technology in areas with limited resources. Consequently, new affordable, highly sensitive, and short-time diagnostic methods are urgently needed to improve the outcomes of TBM.

We compared confirmed or probable BM patients with TBM patients for the following reasons: first, patients with BM were usually difficult to distinguish from patients with TBM. High protein and low CSF glucose or low CSF glucose (<50% of that in blood) were usually found in both patients. In present study, the normal range of CSF glucose was present in only 25 (10%) patients and the normal range of CSF protein was present in only 5 (2%) patients. Furthermore, we found that 21 (21%) patients with BM had a predominant lymphocytic response in CSF, wherein 15 had accepted intravenous antibiotics before admission. This was much higher than the other report [19], and such cytological manifestations can cause a lot of confusion in the initial diagnosis. Second, both groups of patients needed prompt diagnosis and treatment to save lives. In addition, the etiological diagnosis of both groups was all difficult. Only 50% of TBM patients and 20% of BM patients were definitely diagnosed in this research. What is worse is that if the CSF examination was conducted after antibiotics, the chance to identify an organism might be reduced by 44% [20, 21]. Therefore, it is even more difficult to distinguish TBM patients from patients with partly treated BM.

Different studies have been objected to distinguish between TBM and BM depending on clinical data and laboratory features according to limitations of these diagnostic techniques. Thwaites and colleagues employed 143 cases with TBM and 108 cases with BM in Vietnam to develop a scoring system in the light of clinical and laboratory features. It was found that five features, including age, disease course, blood white cell count, total CSF white cell count, and neutrophil proportion in the CSF, were independently correlated with TBM in a multivariate logistic regression. A diagnostic rule from these features had 97% sensitivity and 91% specificity [6]. This diagnostic rule was validated in different populations and settings and revealed with 90% sensitivity and 50–90% specificity [22–26]. Unfortunately, the diagnostic scoring system was found to be less effective when some partially treated BM were encountered. In Turkey [7], the serum C-reactive protein (CRP) level is regarded as a new diagnostic index. A sensitivity of 95.5% and a specificity of 100% were found in the modified diagnostic rule. In Morocco [8], the study found that the female gender and focal deficits were also independent predictors of TBM and developed a simple diagnostic rule for TBM. The study proved that the sensitivity and specificity of the diagnostic rule tend to be 87% and 96%, respectively. The performance of these diagnostic rules was variable in different settings and populations; therefore, we attempted to establish our own diagnostic scoring system to be a diagnostic aid for TBM in China.

In this work, the univariate analysis of admission variables revealed some clinical and laboratory features that were potentially discriminative. Patients with TBM presented with earlier incidence. They have a higher probability to develop symptoms of TB poisoning and cranial nerve palsies, and they usually suffer from hyponatremia; their CSF tends to be clear, with moderate neutrophils and lymphocytes, as well as a decrease of CSF chloride. In this context, 19 (13%) TBM patients had cranial nerve involvement. 12 patients had abducent nerve (sixth cranial nerve) palsy; 3 patients suffered from oculomotor nerve (third cranial nerve) palsy; 2 patients were diagnosed as optic nerve (second cranial nerve) palsy, and 2 patients had facial nerve (seventh cranial nerve) palsy. Available studies suggest that approximately one-quarter of TBM patients suffer from cranial nerve involvement; it should be noted that the abducent nerve is the most frequently involved nerve [1]. Having thick gelatinous exudates in the basilar regions of the brain is the pathological feature of TBM. And cranial nerves are affected either due to entrapment of the nerve trunk in thick basilar exudates or intracranial pressure increase [27]. The cranial nerve palsies are a characteristic manifestation of TBM, although this variable does not present in the final diagnostic model. A multivariate logistic regression was applied for modeling of five characteristics that are independently predictive of TBM. From these characteristics, a diagnostic rule was created to distinguish TBM from BM: TDI = DI (disease course of more than 4.5 days) + DI (white blood cell count of less than less than 12.15 × 10^9^/L) + DI (serum sodium of less than 132.8 mmol/L) + DI (total CSF white cell count of less than 499 × 10^3^/mL) + DI (the neutrophil proportion in CSF of less than 59%). A segmentation of 6 in the ROC analysis was selected because it shows the greatest sensitivity (87%) and acceptable specificity (94%).

The parameter of the serum sodium level was included to our diagnostic formula. In this study, 103 (73%) patients with TBM had hyponatraemia (plasma sodium < 135 mmol/L) and 26 (18%) patients were classified as profound hyponatraemia (plasma sodium < 125 mmol/L). In the Vietnam diagnostic rule, this parameter was excluded because of massive missing values in that study. In the patients with TBM, hyponatremia may occur with a higher frequency than other CNS infections due to ventriculitis, leptomeningeal inflammation, raised intracranial pressure, and hydrocephalous [28]. Approximately 40–50% of patients with TBM suffer from hyponatraemia. The most possible reasons of hyponatraemia of patients with TBM include syndrome of inappropriate secretion of antidiuretic hormone (SIADH) and cerebral salt-wasting syndrome (CSW) [29]. However, the mechanism of hyponatraemia remains unclear and the distinguishing between the two conditions is very difficult. We found that hyponatraemia was independently predictive of TBM.

The study shows that simple clinical and basic laboratory parameters can be applied to distinguish TBM from BM patients and we propose a diagnostic scoring system with an 87% sensitivity and a 94% specificity. Some important limitations in this study still need to be solved. First, this paper is about a retrospective study; therefore, some features were inaccessible. Second, cerebral imaging had not been included in the diagnostic rule, because cerebral imaging was not made in 13% (*n* = 19) of TBM and 20% (*n* = 20) of BM cases. Third, 114 of 241 patients accepted tests about antibodies to HIV and only one with TBM was positive. Therefore, as for areas with a high prevalence in acquired immune deficiency syndrome (AIDS), the diagnostic scoring system is not recommended.

In conclusion, the diagnostic scoring system proposed by the author in this study can help the physicians who can do empiric diagnosis of TBM in a short period and prompt antituberculous therapy in areas with tuberculosis high incidence, especially with the condition of limited microbiological resources. Further research is needed to validate the diagnostic scoring system.

## Figures and Tables

**Figure 1:** Receiver operating characteristic (ROC) for prognostic indexes from the logistic regression model.

**Table 1:** Diagnostic criteria about the classification of definite, probable, and possible tuberculous meningitis.

	Score	Definite TBM (*n* = 141) *n*	Probable TBM (*n* = 44) *n*	Possible TBM (*n* = 99) *n*
Clinical criteria of the maximum score = 6				
Duration of symptom exceeding 5 days	4	138	44	94
Systemic symptoms about tuberculosis (one or more of the following): weight loss (or poor weight gain in children), night sweats, or persistent cough for over 2 weeks	2	32	18	4
Recent (within a past year) close contact history with an individual with pulmonary tuberculosis or positive TST or IGRA (only children < 10 years old)	2	0	0	0
Focal neurological deficit (excluding cranial nerve palsy)	1	12	4	5
Cranial nerve palsy	1	19	6	4
Disturbance of consciousness	1	66	21	11
CSF criteria with a maximum score = 4				
Clear appearance	1	120	36	92
Cells: 10–500/*μ*L	1	131	41	88
Lymphocytic predominance (>50%)	1	115	41	74
Protein concentration > 1 g/L	1	121	38	47
Ratio between CSF and plasma glucose < 50% or an absolute CSF glucose concentration < 2.2 mmol/L	1	116	39	27
Brain imaging criteria, maximum score = 6				
Hydrocephalus	1	26	6	3
Basal meningeal enhancement	2	51	19	4
Tuberculoma	2	56	16	4
Infarct	1	26	11	6
Precontrast basal hyperdensity	2	4	0	0
Evidence of other tuberculosis, maximum score = 4				
Chest radiograph showing active tuberculosis: tuberculosis index = 2	2	70	25	6
Chest radiograph for active tuberculosis: miliary tuberculosis signs = 4	4	23	7	0
CT/MRI/ultrasound results about tuberculosis outside the CNS	2	20	5	2
AFB identified or *Mycobacterium tuberculosis* from another source(i.e., sputum, lymph node, gastric washing, urine, and blood culture)	4	6	2	0
Commercial positive *M. tuberculosis* NAAT from extraneural specimen	4	0	0	0

TBM: tuberculous meningitis; TST: tuberculin skin test; IGRA: interferon-gamma release assay; CSF: cerebrospinal fluid; CNS: central nervous system; CT: computed tomography; MRI: magnetic resonance imaging; AFB: acid-fast bacilli; NAAT: nucleic acid amplification test.

**Table 2:** Univariate analysis for the comparison of variables between tuberculous meningitis patients and bacterial meningitis patients.

	Tuberculous meningitis		Bacterial meningitis		*P*
	Median (IQR) or *n* (%)	*n*	Median (IQR) or *n* (%)	*n*	
Age (years)	35 (23–51)	141	30 (24–46)	100	0.198
Male (sex)	83 (59%)	141	72 (72%)	100	0.036
Disease course (days)	14 (7–28)	141	3 (1–6)	100	≤0.001
Headache	129 (92%)	141	91 (91%)	100	0.895
Fever	128 (91%)	141	95 (95%)	100	0.220
Nausea	99 (70%)	141	65 (65%)	100	0.393
Vomiting	96 (68%)	141	61 (61%)	100	0.256
Coma before admission	66 (47%)	141	50 (50%)	100	0.626
Psychiatric symptoms	46 (33%)	141	39 (39%)	100	0.308
Seizure	23 (16%)	141	14 (14%)	100	0.624
Meningeal signs	104 (92%)	141	92 (92%)	100	≤0.001
Cranial nerve palsies	19 (14%)	141	3 (3%)	100	0.006
Focal neurological deficit	12 (9%)	141	3 (3%)	100	0.082
Coughing for 2 or more weeks	15 (11%)	141	5 (5%)	100	0.059
Recent loss of weight	19 (14%)	141	0	100	≤0.001
Night sweats	15 (11%)	141	1 (1%)	100	0.003
BMRC TBM grade					0.265
Stage I	11 (8%)	141	6 (6%)	100	
Stage II	47 (33%)	141	44 (44%)	100	
Stage III	83 (59%)	141	50 (50%)	100	
Hemoglobin (g/L)	130 (119–139)	141	135 (123–144)	100	0.108
HCT %	38 (35–39)	141	39 (36–42)	100	0.009
WBC count (10^9/^L)	9 (6–11)	141	17 (13–21)	100	≤0.001
Blood % neutrophils	80 (74–85)	141	88 (81–92)	100	≤0.001
Serum sodium (mmol/L)	131 (125–135)	141	139 (134–142)	100	≤0.001
CSF opening pressure (mm H_2_0)	295 (210–350)	141	272 (203–309)	100	0.321
Clear CSF appearance	120 (85%)	141	27 (27%)	100	≤0.001
CSF total WCC (10^3^/mL)	150 (60–300)	141	1145 (489–3160)	100	≤0.001
CSF % neutrophils	15 (10–30)	141	80 (60–90)	100	≤0.001
CSF protein (g/L)	1.55 (1.12–2.08)	141	1.65 (1.14–2.82)	100	0.102
CSF/blood glucose	0.35 (0.23–0.46)	141	0.29 (0.08–0.39)	100	≤0.001
CSF chloride (mmol/L)	111 (106–118)	141	117 (111–123)	100	≤0.001

IQR: interquartile range; BMRC: British Medical Research Council; TBM: tuberculous meningitis; CSF: cerebrospinal fluid; WBC: white blood cell; WCC: white cell count.

**Table 3:** Original multivariate logistic regression analysis.

	*β*-Coefficient	Odds ratio (95% CI)	*P* value
Disease course	−0.088	0.916 (0.859–0.977)	0.007
WBC count	0.191	1.211(1.046–1.402)	0.010
Blood % neutrophils	−0.081	0.922 (0.869–0.979)	0.008
Serum sodium	0.125	1.133 (1.021–1.257)	0.019
CSF total WCC	0.001	1.001 (1.000–1.002)	0.024
CSF % neutrophils	0.022	1.022 (1.005–1.04)	0.011

WBC: white blood cell; CSF: cerebrospinal fluid; WCC: white cell count.

**Table 4:** Multivariate logistic regression analysis about the converted categorical variables.

	*β*-Coefficient	Odds ratio (95% CI)	*P* value
Disease course of more than 4.5 days	2.239	9.384 (2.714–32.447)	≤0.001
WBC count of less than 12.15 × 10^9/^L	2.318	10.157 (3.134–32.916)	≤0.001
Serum sodium of less than 132.8 mmol/L	1.163	3.200 (1.089–9.407)	0.034
CSF total WCC of less than 499 × 10^3^/mL	2.586	13.278 (4.222–41.756)	≤0.001
CSF % neutrophils of less than 59%	1.365	3.916 (1.423–10.779)	0.008

WBC: white blood cell; CSF: cerebrospinal fluid; WCC: white cell count.

**Table 5:** Weighted diagnostic index of clinical variables in the diagnostic rule.

Clinical variables	Diagnostic index
Disease course (days)	
>4.5	2
≤4.5	0
WBC count (10^9/^L)	
>12.15	0
≤12.15	2
Serum sodium (mmol/L)	
>132.8	0
≤132.8	1
CSF total WCC (10^3^/mL)	
>499	0
≤499	3
CSF % neutrophils	
>59	0
≤59	1

WBC: white blood cell; CSF: cerebrospinal fluid; WCC: white cell count.

## Data Availability

All data generated or analyzed during this study are included in this article.
